The article "Analysis of Performance Improvement of Real-time Internet of Things Application Data Processing in the Movie Industry Platform" was published in 2022. Journal: Comput Intell Neurosci.

# Analysis of Performance Improvement of Real-time Internet of Things Application Data Processing in the Movie Industry Platform

**DOI:** 10.1155/2022/5237252

**Published:** 2022-10-10

**Authors:** Yang Meng

**Affiliations:** ^1^Macau University of Science and Technology, Faculty of Humanities and Arts, 999078 Macau, China; ^2^Communication University of Shanxi, Shanxi 030619, China

## Abstract

The goal of this study is to plan and develop complete strategies to improve the performance of film industry. The primary objectives of this study are to investigate a dataset generated by a IoT application and the nature of the data forms obtained, the speed of the data arriving rate, and the required query response time and to list the issues that the current film industry faces when attempting to handle IoT applications in real time. Finally, in film industry platforms, high performance with varied stream circulation levels of real-time IoT application information was realized. In this study, we proposed three alternative methods on top of the Storm platform, nicknamed Re-Storm, to improve the performance of IoT application data. Three different proposed strategies are (1) data stream graph optimization framework, (2) energy-efficient self-scheduling strategy, and (3) real-time data stream computing with memory DVFS. The work proposed a methodology for dealing with heterogeneous traffic-aware incoming rate of data streams Re-Storm at multiple traffic points, resulting in a short response time and great energy efficiency. It is divided into three parts, the first of which is a scientific model for fast response time and great energy efficiency. The distribution of resources is then considered using DVFS approaches, and successful optimum association methods are shown. Third is self-allocation of worker nodes towards optimizing DSG using hot swapping and making the span minimization technique. Furthermore, the testing findings suggest that Re-Storm outperforms Storm by 20–30% for real-time streaming data of IoT applications. This research focuses on high energy efficiency, short reaction time, and managing data stream traffic arrival rate. A model for a specific phase of data coming via IoT and real-time computing devices was built on top of the Storm platform. There is no need to change any software approach or hardware component in this design, but only merely add an energy-efficient and traffic-aware algorithm. The design and development of this algorithm take into account all of the needs of the data produced by IoT applications. It is an open-source platform with less prerequisites for addressing a more sophisticated big data challenge.

## 1. Introduction

Digital technology is altering scientific practice. Digital imagery, sensors, analytical apparatus, and other techniques are becoming increasingly important in many areas of science for experimental and observational study. Usually big data is one of the technologies to deal a massive number of datasets [1, 2]. Currently, two different processing/computing platforms are there to deal big data. One is a batch computing platform like Hadoop. The second one is stream computing like Storm. Because it takes data in a stream form from collections of hardware or software sensor and computes continuous time data streams, stream processing is a key feature of this program on real-time online high-speed streaming data. For processing enormous volumes of streaming data, real-time stream computing is required. The future consignment is based on common task structure experiential in several Internet of things (IoT) fields for decision-making in real time, and the input data streams are obtained from real IoT applications observations from various applications like smart hospitals, smart cities, and entertainment like film industry. The collaboration of this application is full by the integration of business, consumer, and business and industry Internet access, and industrial IoT consumer interactions is used by IoT applications [3–5].

The article "Analysis of Performance Improvement of Real-time Internet of Things Application Data Processing in the Movie Industry Platform" was published in 2022. Journal: Comput Intell Neurosci.

In big data systems, the preparation of high-speed continuous information in stream processing required for processing is also a noteworthy goal. In the fault-tolerant population-stream registration programming mentioned by Neumeyer and Robbins(2010), which mimics S4, the shortcomings of group processing are addressed by equal-flow computation with low inertia and acceleration, but the full-population-stream processing of both platforms has drawbacks. By conducting a thorough examination of existing rules, it was discovered that the present film and television engines are not meeting the demands of IoT data streams. Unknown energy consumption, reaction time period, and traffic velocity data entering the streaming data engine are provided by the IoT data element. IoT is expanding and making immense measures of constant information; it is a major testing assignment in IT industry. Stream registering is reasonably the quickest and most proficient answer for getting profitable data from enormous information. In addition, numerous information streams from divergent information sources may shape a mix of the information sorts that might be inconsistent [6–8].

The goal of this study is to plan and develop complete strategies to improve the performance of film industry. The environment for IoT application datasets makes a platform towards using data stream optimization, energy-efficient data stream dynamic scheduling, and memory DVFS approaches to reduce energy consumption. Future IoT advancements will handle highly dispersed IoT applications that necessitate a high level of distribution and process at the network's edge by using platform that would provide compute, storing, and data networks between edge devices or computing data centers. These systems will enable emerging Internet of Things applications that require real-time latency. This study effort begins by outlining the mathematical relationship between energy use, reaction time, and overall asset use in the film business. It finds out how to satisfy the reduced response time and the high energy efficacy targets, displaying DSG in film industry conditions by alluding to the appropriated stream figuring hypotheses, distinguishing that the vertices weight are vertices in DSG, and achievement energy utilization of a distribution conspire for a DSG at a particular information stream speed, and doling out assignments by the energy proficient heuristic movement mindful planning strategies.

The article "Analysis of Performance Improvement of Real-time Internet of Things Application Data Processing in the Movie Industry Platform" was published in 2022. Journal: Comput Intell Neurosci.

The study's goal is to increase the performance of real-time IoT data processing on a film industry framework. The main goals of this research are to evaluate a dataset generated by a popular IoT application and the nature of the information obtained, the velocity of responsive service rate to computing, the query-processing time needed, and to list the issues that the current film industry system faces when dealing with IoT applications in real-world time. The high performance of real-time iot application information with different flow circulation degree is realized on the film industry platform.

## 2. Methods

### 2.1. Data Stream Graph Optimization Framework

Approaches to constructing a BDSC platform based on the data streams graph optimization method make it possible to optimize DSG via critical route removal and parallelism. Optimizing an application's scheduling strategy DSG to assets is being considered, but how to progress the DSG is being disregarded. To attain high consistency, it is critical to first obtain a good image of the altered state of the DAG and then select which vertex of a DAG should indeed be rescheduled. Before submitting the graph to the Storm stage, the client plans the structure of the DSG based on the capability of the application. To ensure high stability, establish a fair picture of a DAG's changing state before deciding which vertex of the DAG must be rescheduled. More crucially, understanding how to boost framework strength while assuring makes span reduction and controlling superior, and response time trade off in a productive and practicable method is required, which is absent in the bulk of current scientists in BDSC situations [9–12].

The article "Analysis of Performance Improvement of Real-time Internet of Things Application Data Processing in the Movie Industry Platform" was published in 2022. Journal: Comput Intell Neurosci.

#### 2.1.1. System Architecture

The four stages of the Storm computing platform are responsible for real-time data streaming (Figure 1) which are task assessment, scheduling phase, processing phase, and storage area. It demonstrates DSG optimization utilizing two unique strategies: critical route elimination, which avoids the crucial route to modify the latency of the produced data stream, and data stream parallel processing, which approaches heavy nodes of the are computing data stream operating in parallel (Figure 1).

#### 2.1.2. Experimental Set-Up

A model resolve is the process of creating a simulation environment for real-time computing. To create a simulation environment, hardware requirements are utilized. To test the efficacy of the suggested paradigm, an experimental setting with high-speed network access was created. Intel i7 CPU, 16 GB RAM, 1 Gbps network access, and 104 core workstations were used to evaluate the suggested concept. Two proposed methodologies were applied to tuples that comprised a stage of the Storm framework. Ubuntu server 14.01, Storm 0.10.0, Java 1.8.25, Zookeeper 3.4.0, and Python 3.0 are the software requirements for computing the results. A cluster's performance is evaluated using real-world data tests. The cluster comprises of 18 computers, one of which is assigned as a main node that runs Storm Nimbus, one as a Zookeeper node, and the remaining 16 as subnodes. Each computer runs with Linux Ubuntu Server 13.04 and is equipped with twin 8-core Intel Core (TM) i7-4790 processors running at 3.6 GHz, 16 GB of memory, and 1 Gbps NIC (Figure 2).

#### 2.1.3. Optimizing

Before the graphs have been submitted to the phase on the Storm platform, the client defines the structure of the DSG based on the capacities of the application [13]. DSG has two variables such as *G* = (VG, EG); in this group, the vertex is treated as DAG, which is a consequence by the DAG. Each *G* continues using two parameters *G* = (VG, EG), where VG is a group vertex and EG is a group edge, and subgraph Gs, ∀ Vi *ϵ* VGs than ∀ VG *ε* VGs, the way it is travelling the DAG route. If S ≠ E, then the starting and ending points of a (Vs, Ve) are the same, the graphs are not directed, and it usually indicates a null vertex/node. Topological sort (TS) is also another type of graph that does not have cycle structures. DAG stands for topology sort order. The DAG considers partitioning a graph based on TS by separating the vertex of a graph. A partition graph (GP) is a topology-based partitioning vertex graph GP = {GP1, PP2, PP3 … . .}. For each partition, GP1 = {v1, v2, v3,… } ∈ G and GP2 = {v1, v2, v3,… } ∈ *G*. It is a subgroup containing ∀ *i* ≠*j* i, *j* ∈ (1, n), then GPi ∪ GPj = ∅ ⋃ GPi ≠ n 1 VG and *G* = (VG, EG). Each vertex and edge contains some tuples VG = (idv, fv, cvi, v, ov) and EG = (ide, ce) P(Vs, Ve), where graph vertices = {V1, V2, V3,… … … Vi}, graph edges = {E1, E2, E3,… … … Ej}, start vertex and end vertex = Vs, Ve identification of vertices, function, computing cost, data input streams, output data stream idv, fv, cv, iv, ov 52 ide, Ce = directed edge identification, directed edge communication cost. In the graph shown in Figure 2 , it starts vertex from V1 and ends at V8, and it is not encompassing circles and it *ϵ*G {V1, V2, V3, V4, V5, V6, V7, V8}, and in this one subgraph, we assume, for example, {V1, V3, V5, V6, V8} ∈ G, and there are two routes in this above graph {V1, V2, V4, V7, V8} and {V1, V3, V5, V6, V8} ∈ *G*. Furthermore, TS is depicted in the graph (Figure 2).

The article "Analysis of Performance Improvement of Real-time Internet of Things Application Data Processing in the Movie Industry Platform" was published in 2022. Journal: Comput Intell Neurosci.

### 2.2. Energy-Efficient Self-Scheduling Strategy (EESSS)

#### 2.2.1. Framework

In Storm processing area, the model for observing digital streaming graph, optimization model for DAG, adaptive streaming data deviation model, energy-aware scheduling of DAG approach, and traffic-aware resource rescheduling method for the DAG model work to care for constant traffic rate for scheduling intends on top of the open-source Storm platform. The storm is indeed a BDSC system that is distributed. To disperse data streams between several instances of a vertex, the energy-efficient traffic awareness resource scheduling paradigm is employed. The DAG-based energy-aware scheduling approach is utilized to give a DAG self-scheduling strategy based on traffic rate that is created by a user and is in a traffic rate stream. The DAG model's traffic awareness based resource rescheduling is used to reschedule a DAG in an energy-efficient manner and to achieve high energy efficiency in a constant fashion [14–18] (see Figure 3).

#### 2.2.2. System Architecture

The flow of system is considered either by user or hardware generation of data streams as well as its formation as a graphical form, and then it is transmitted by the Storm computation, and this process using predefined task scheduling by round Robin made reference from Zong et al. for enhancing the performance of standard scheduling strategic approach which is amended as an energy-efficient traffic-aware resource allocation method (as shown in Figure 4) [18].

#### 2.2.3. Experimental Set-Up

By changing the default scheduling method in Storm's IScheduler surface and gaining correct results, efficient energy self-scheduling methods are used to improve performance (by optimizing energy efficacy and reducing reaction time through varied levels of traffic of the data streams). The Storm platform simulation environment is built in fully functioning parallelism, fault tolerance, and distribution of the latest version of software, i.e., Storm 0.10.0. A 4 core Intel 13 processor 2.00 GHz 64 Bit CPU, 16 GB memory, and 512 Mbps network access are required for virtual machines. 4 core two PCs, each with a 10 TB external storage capacity, are joined together. A Linux server is installed on each system (Ubuntu version 14.01). The software components listed below are often built and used in combination with Java 1.8, Zookeeper 3.4.0, and Python 3.0. Furthermore, on the Storm platform, all upgraded scheduling techniques replace the default scheduling approach with improved and efficient traffic-aware scheduling for energy. In Storm UI, the output is being watched. For performance purposes, the average tuples computation is employed. This used Storm's default timing technique to measure the process time of every tuple. Storm UI can gather such information, but then it only displays the 10 minute average. According to Zhao Zhibin et al., the recommended approach trial and execution takes about one minute rather than averages, providing us with far more precision in real-time performance estimate (2008). During the investigation, Ubuntu Linux used the NTP protocols standard to synchronize worker nodes [19].

The article "Analysis of Performance Improvement of Real-time Internet of Things Application Data Processing in the Movie Industry Platform" was published in 2022. Journal: Comput Intell Neurosci.

### 2.3. Real-Time Data Stream Computing with Memory DVFS

DVFS is a popular technology to scale voltage frequency according to the application precedence at the CPU level. In this work, this technique is apllied to the memory level to reduce energy consumption and improve performance.

#### 2.3.1. Experimental Set-Up

Adding frequency scaling-based control algorithm for improving energy efficiency is done. It minimizes the application's energy usage while increasing its efficiency. The frequency-based control mechanism is software-based.  Figure 5 depicts the data stream control method. It is to handle the large data stream computing environment while processing data from IoT applications. It experiences difficulties; thus, it is searching for more gap filling to assist it in overcoming these difficulties. The Storm framework in the stream computing is open source and is developed to address the most pressing demands of the current streaming data component. The scheduling mechanism used in this one is Round Robin by default. It is undesirable as data transmission is rather high at the slow point, and energy usage is quite significant for that reason. Data were generated by devices (Figure 5).

#### 2.3.2. Optimization

Sun et al. used the DVFS approach to the enormous data leaking group and scientific proof presented with each on/off chips doling out workloads [20]. The load of an errand is defined as the total of the CPIs of all bearings further towards the path stream of the venture. A variety of component factors influence the task load, including the on-chip halt cycle number owing to data reliance or the branched miss forecast, and the off-chip log jam phase checks due to I/*D* TLB miss or I/*D* store miss. The CPU waits until the requested memory exchange is accomplished during an off-chip access. As a result, the processor clock cycle during an off-chip is altered. To comprehend the load rot framework, a few definitions are required.

The article "Analysis of Performance Improvement of Real-time Internet of Things Application Data Processing in the Movie Industry Platform" was published in 2022. Journal: Comput Intell Neurosci.

**Definition 1 .**

Won is the number of clock cycles necessary for the CPU to complete the set of on-chip instructions, which are made entirely of the CPU. The performance time required to complete Won, *T* on, fluctuates according to CPU frequency, *f* cpu, and is calculated as *T* on = Won/*f* cpu.

**Definition 2 .**

Woff is the number of external clock cycles required to conduct the set of off-chip accesses. It is worth noting that the CPU delays until the peripheral memory operations are completed. The execution time necessary to complete Woff, *T* off, is computed as a function of the outward memory clock cycle frequency, *f* ext as *T* off = Woff/*ft* = −logf (*T* o *f* 2 Wo *f* 2) ex, *x* ≠ 0 and −Wo *f* 2 ≠ 0 ∅, *x* = 0 and −Wo *f* 2 ≠ 0 and −logf (*T* o *f* 2 Wo *f* 2) ≠ 0 *t* ∈ ℝ, *x* = 0 and −logf (*T* o *f* 2 Wo *f* 2) = 0 and −Wo *f* 2 ≠ 0. Based on defined in equations 5.1 and 5.2, Won and Woff is written as Won = *N*.CPUIavg on and Woff = *M*. CPI off avg (5.1), where CPI avg on represents the average number of CPU clock pulses per on-chip instruction, *M* represents the number of off-chip access, and CPI avg off represents the average of external clock cycles per off-chip access. The execution time, *T*, for a job is determined using these two definitions as *T* = *T* on + *T* off = *N*.CPUIavg on fcpu + *M*. CPI off avg fext (5.2) When the CPU frequency changes, the change in *T* is solely due to *T* on (∆T ∆f CPU) = ∆T on ∆f cpu, ∆T off ∆f cpu 0 (5.3) Lemma 1: Each degree of energy consumption is based on computing each job and reaction time based on a scheduling element, and two tasks A and B are considered. Proof: Assume 89 Accept to make a change in which you have two distinct ideal schedules A and B. Consider a third schedule U wherever for all the tasks *i*, xi(U) = (xi(A) + xi(B))/2. Now privilege that F(U) ≤ (F(A) + F(B))/2 = F(A) = F(B) and E(U) < (E(A) + E(B))/2. As a result, neither S nor *T* are optimal for one may enhance the plan by investing A − E(U) energy into occupation *n* in U to show evidence of better reaction time than F(U). This opposes the model of S. To demonstrate F(U) ≤ (F(A) + F(B))/2 = F(A) = F(B), consider a certain task *b*. Then there is some work “a” Cy (U) = rx + ∑ (U) *yi* = *a*. So by the description of U, Cy(U) = rx + ∑(xi(A) + xi(B))/2y *i* = *x*. But in S, let it necessarily be the case that Cb (*A*) ≥ ra + ∑ (xi (*A*) *yi* = *x* (5.4). For A, must procedure jobs *x* finished *y* among response time rx and Cy(A). Similarly, Cy (B) ≥ rx + ∑ xi(B) *y i* = *x* (5.5). By taking the average of these two equations, (Cy(A) + Cy(B))/2 ≥ ra + ∑ (xi (*A*) + xi(B))/2 y*i* = *x*. (5.6). The right-hand side of this inequality is precisely Cy (U) in this processing. Hence, (Cy(A) + Cy(B))/2 ≥ Cy(U). Because *y* was picked at random, it follows that F(U) ≤ (F(A) + F(B))/2. Note that the function f(*x*) = 1 x *α*−1 is a rounded function when *α* > 1, and *f* (*x* + *y* 2) < (f(*x*) + *f*(y))/2. It thus immediately follows E(U).

The article "Analysis of Performance Improvement of Real-time Internet of Things Application Data Processing in the Movie Industry Platform" was published in 2022. Journal: Comput Intell Neurosci.

## 3. Results and Discussions

All of the findings are obtained from various sources in order to verify the working nature of the offered technique. Streams submitting at various traffic levels are on top of it, testing to see if it is appropriate for all situations and comparing the findings to different qualities. The principal input type is data generated by IoT devices, which is perfect for sampling real-time and high-velocity data but also a difficult task in today's IT industry. The proposed method is for efficiently providing greater control over IoT-related data processing via big data platforms which meets this aim, meaning that it is suitable for readily computing various types of high-velocity data.

In this paper, we presented a new application standard to measure BDSC in the IoT environment. Data phases, like stream processing system (SPS), are required for IoT applications' high speed control needs, and recommended work overload calculates their viability using basic tasks found in IoT applications, as well as entirely practical implications for the fact-based outline and predictive investigative process. These are combined with two trustworthy information sources from the urban IoT testing and transportation businesses. The proposed standard for the widely used Apache Storm SPS, as well as the implementation steps, has been accepted. A task scheduling planning calculation for managing massive data streams in mobile Internet service is provided to establish parallel machine execution, and the streaming query graph is functioned to determine each edge weight. The remodeling findings show that using the appropriate number of logic machines reduces the response time of framework substantially, and scheduling several tuples at once reduces framework connection switching. The calculating approach used in this study can increase the productivity of massive data stream processing in portable one. The suggested data stream optimization has indeed been accepted as the benchmark for the widely used Apache Storm SPS and the execution methods introduced. A dynamic programming planning calculation for big data stream handling in mobile Data Internet access is offered to create parallel machine execution, and the streams query graph is worked to determine each edge weight. The remodeling findings show that using the appropriate number of logic machines reduces framework response time substantially, and scheduling several tuples in one go minimizes framework connection switching. This study's calculation has the potential to increase the efficiency of enormous data stream handling in mobile Internet access. Reduced scheduling rates, on the other hand, will lead to IoT implementation [21–25].

The article "Analysis of Performance Improvement of Real-time Internet of Things Application Data Processing in the Movie Industry Platform" was published in 2022. Journal: Comput Intell Neurosci.

### 3.1. Energy-Efficient Self-Scheduling Strategy (EESSS)

All of the findings are collected from various sources in order to verify the effectiveness of the suggested approach, with streams submitting at various traffic levels on top of it, testing to see if it is appropriate for all situations and comparing the findings to different qualities. The principal input type is IoT-produced data, which is appropriate for sampling real-time and high-velocity data but also a difficult task in today's IT industry. The proposed method is for efficiently providing improved control for Internet-of-things data computing by using big data frameworks that meets this aim, meaning that it is suitable for readily computing various types of high-velocity data. Obtaining data samples of real-time IoT creation from Shahrivari's CityPulse Database Collection (2013). There are several types of datasets accessible, such as pollution, weather, and road traffic which developed a virtual environment for controlling data speed with various traffic mediums.

When compared to the present model, evaluating the suggested model with appropriate varied traffic mediums would yield better performance. First, allocating a low traffic medium, then making numerous alterations and eventually achieving peaceful outcomes in all aspects. Those graphs are provided below. We improved energy economy and reduced reaction time by varying the traffic volumes of information streams. The graphs show the outcomes of how to use energy at the system level while lower traffic levels are evaluated. Figure 4, 6 depicts a 0–250 tuple which constructed a variable of tuples on submitting somewhere in the middle of the range at the responding time and energy consumed with both platforms under the identical circumstances. Re-Storm outperforms both Storm and Re-Storm in all scenario test situations, demonstrating that it is well suited for IoT-sensing data. Online ongoing information is indistinguishable, divergent arriving rate, and it does not have a consistent activity detecting medium. It was examined what all significance are there for upgrading stream diagrams and energy proficiency requirements for BDSC condition. The proposed approach considered two variables for enhancing their execution proficiency. Initially, it is adjusting their planning system with unessential activity stream support, and second is enhancing their diagrams utilizing basic way disposal to keep up a voting demographic for various movement medium information, besides, updating 20–30% proficiency in stream figuring. At long last, it makes a colossal effect on general all BDSC condition obtaining exceptional performance throughout the whole big data platform, with a focus on real-time as well as IoT information. This research concentrates on improving energy efficiency, fast reaction time, and controlling the arrival rate of data stream traffic. On top of the Storm system, a model for a specific phase of data arriving from IoT and real-time computing was built. This design does not require any changes to the software or hardware; simply add an energy-efficient and traffic-aware algorithm. The design and development of this algorithm take into account all of the needs of the data produced by IoT applications. It has less prerequisites for dealing with a more complicated big data challenge and is an open-source system [26, 27].

The article "Analysis of Performance Improvement of Real-time Internet of Things Application Data Processing in the Movie Industry Platform" was published in 2022. Journal: Comput Intell Neurosci.

### 3.2. Real-Time Data Stream Computing with Memory DVFS

This approach presented the essential tradeoffs in memory recurrence scaling and played out an underlying assessment utilizing a straightforward and natural calculation. However, more work stays to be finished. To begin with, a basic system and a vast plan space, both plays a role in measuring and anticipating the effect on execution and on expecting the future effect of memory recurrence changes. Additionally, work can explore both the estimation and forecast parts of this issue and portray how different sorts of workloads react to expanded memory inertness. This paper also examined the interaction between memory storage scaling and CPU voltage or frequency scaling (DVFS). Positively, the two devices could exchange signals. It is also possible that higher productivity gains are possible under combined control as when the two work independently. At long last, it is thought to be just SPEC CPU2006 in this work; assist assessments are important to evaluate execution affect in different workloads. In this paper, a model was suggested to analyze memory frequency/voltage scaling in order to maximize energy efficiency and minimize memory power. We describe a control technique that decreases memory frequency while reducing performance effect, based on the fact that a large amount of memory system power is frequency dependent. The essential discovery is that changing memory frequency has no effect on memory access latency when memory bandwidth usage is low. By monitoring memory bandwidth consumption, the suggested control method raises memory frequency when utilization exceeds a certain threshold, hence limiting the performance effect. In this way, DVFS can be a useful energy-saving solution, especially when memory bandwidth consumption is modest [28].

## 4. Conclusion, Future Work, and Significance of the Contribution

### 4.1. A Data Stream Graph Optimization Framework

It maintains a consistent high efficiency and a short response time. It decreases the utilization no. of computing nodes. The quantification of distribution scheme for a DSG is energy efficient at a given information stream velocity and merging of heavily weighted vertices on large DAG to perform logical splitting to maximize the energy efficiency, altering their scheduling strategy with inappropriate traffic streams and optimizing DSG using vertices weight-based exclusion. Moreover, the upgrading approach against the existing platform enhanced efficiency shown by 20–30%. Finally, it makes a huge effect on the whole BDSC environment.

### 4.2. An Energy-Efficient Self-Scheduling Strategy

This technique presents Re-Storm, a revised Storm streaming engine, as well as an energy-aware stream congestion consolidation mechanism for allocation of resources. As per the arriving size of the data stream weight of each vertex, it should allocate resources as per online data stream traffic rate. Finally, achieving low response time and high energy efficiency with dissimilar traffic levels of streams in BDSC is called as Re-Storm.

### 4.3. Real-Time BDSC Platforms towards Improving Efficiency

A new main memory-based control algorithm strategy is proposed for observing memory bandwidth based on task strength adjusting, utilizing its frequency/voltage scaling to minimize performance impact. The power consumption of memory is a significant module of system power. Reduce power consumption memory level as it has high effect and impact on the overall memory level computation system performance. About19% of average gain is achieved against the existing strategies in the evaluation system. Scaling memory voltage/frequency can reduce power utilized by memory with a minimal system performance effect which yields average system energy with a reduction by 2.4%, achieving 0.4% of average memory power reduction. These three proposed strategies are added into the existing BDSC platform towards improving the efficiency of real-time computing of the IoT Applications.

The article "Analysis of Performance Improvement of Real-time Internet of Things Application Data Processing in the Movie Industry Platform" was published in 2022. Journal: Comput Intell Neurosci.

## 5. Additional Points

The limitations of study is that assignments on web-based advancing and engineering which necessitates for the booking component by reallocating the basic vertices continue the basic way of DSG to limit framework variances and response time and integrate the nonbasic vertex and continuing nonbasic manner to increase energy productivity in order to fulfill short response time and greater energy proficiency. Assessing the short response time and high energy effectiveness objectives in film industry environments was not studied here. As they are simply based on point-by-point presumptions, concentrate on limiting energy utilization, or attempt to adjust energy and execution was also not analyzed in details. All the basic vertices just decide low response time on the basic way.

## 6. Conclusion and Future Direction

The work proposed a methodology for dealing with heterogeneous traffic-aware incoming data rate streams, Re-Storm at multiple traffic points, resulting in a short reaction time and great energy efficiency. It is divided into three parts, the first of which is a scientific model for fast response time and great energy efficiency. Then, distribution of resources considering DVFS methods presents effective optimal association methods and self-allocation of worker nodes. Furthermore, the results of the testing indicate that Re-Storm beats Storm by 20–30% for real-time streaming data utilized in Internet of things. It is not necessary to change any software approach or hardware device in this design; merely add an energy-efficient and traffic-aware algorithm. The design and development of this algorithm take into account all of the needs of the data generated by IoT applications. It has only fewer requirements to address a more complex big data problem, as well as an open-source platform.

The following research includes concerns for BDSC environment features, designs for huge real-time data streamed computing environments, influences on task topological graph with a cycle, and a dynamical extensibility of the various streaming data techniques may be studied further, developing BDSC platforms with high fault tolerance, scalability, throughput, and consistency for structuring such a system in a real-world BDSC context.

The article "Analysis of Performance Improvement of Real-time Internet of Things Application Data Processing in the Movie Industry Platform" was published in 2022. Journal: Comput Intell Neurosci.

## Figures and Tables

**Figure 1:** Computing data stream operating in parallel.

**Figure 2:** Model resolve.

**Figure 3:** Framework.

**Figure 4:** System architecture.

**Figure 5:** System architecture.

## Data Availability

The data used to support the findings of this study are included within the article.
